# Deep Learning-Based Postoperative Recovery and Nursing of Total Hip Arthroplasty

**DOI:** 10.1155/2022/7811200

**Published:** 2022-05-26

**Authors:** Hui-Min Wang, Yong-Pei Lin

**Affiliations:** Department of Orthopaedic, The First People's Hospital of Fuyang, Hangzhou, China 311400

## Abstract

**Objective:**

To develop a deep learning-assisted recovery and nursing system after total hip arthroplasty and to conduct clinical trials in order to verify its accuracy.

**Methods:**

In our study, based on manual labeling, the human hip X-ray image library was established, and the deep neural network based on Mask R-CNN was built. The labeled medical images were used to train the model, providing reference for nursing decision after hip replacement. A total of 80 patients with hip injury from 2016 to 2019 were selected for the study. In our paper, the patients were divided into experimental group and control group. The pertinence and effectiveness of the model for postoperative care were evaluated by comparing the hip pain (VAS index), recovery (Harris score), self-care ability (Barthel index), and postoperative complication rate between the two groups.

**Results:**

The pain and complications in the experimental group were significantly lower than those in the control group, the difference being statistically significant (*P* < 0.05); the recovery of hip joint and self-care ability were higher than those in the control group, the difference being statistically significant (*P* < 0.05); the other differences were not statistically significant (*P* > 0.05).

**Conclusion:**

The application of deep learning method in the rapid nursing after total hip replacement can significantly improve the nursing ability. Compared with the traditional method, it has stronger pertinence, faster postoperative recovery, lower incidence of complications, and greatly improves the postoperative quality of life of patients with hip injury.

## 1. Introduction

Total hip arthroplasty (THA) is a terminal procedure for the treatment of patients with hip disease, in which an artificial prosthesis is attached to the normal bone to replace the diseased joint and restore normal hip function. In recent years, with the acceleration of the pace of life, the aging of the population is increasingly serious, the number of patients with hip injury is increasing, and hip replacement has become a treatment for many middle-aged and elderly patients. However, due to the design of the prosthesis and the increasing of quantity model, preoperative planning more complex and uncertain factors in the operation, cause prosthesis and matching rate is not high, patients often occurs in patients with postoperative complications such as long range, hip instability of lower limb, and the poor quality of life, and giving patients postoperative nursing care of science is of great significance [1].

At present, posthip replacement care is mainly planned according to patients' postoperative performance and doctors' clinical experience. X-ray film is the simplest and most direct method for post-THA evaluation and has been widely used in the observation and treatment of postoperative recovery of patients, though the patient's X-ray film can prevent or treat postoperative complications in the early stage, targeted to help patients relieve postoperative pain and restore normal self-care ability as soon as possible [2].

Deep learning has been widely applied in the field of image recognition in clinical medicine [3]. The hip X-ray of patients with hip lesions has obvious structural characteristics, which is very suitable for image recognition by deep learning. Through training, the model can divide the patient's joint area, accurately identify the patient's prosthetic structure, shape, location, and other key information, predict possible complications, assist doctors to formulate postoperative care plans for patients, and improve the nursing effect [4].

## 2. Methods

### 2.1. Target Location and Segmentation Algorithm Based on Mask R-CNN

#### 2.1.1. Mask R-CNN Construction

Mask R-CNN is improved on Faster R-CNN, which extends the Faster R-CNN by adding a branch to predict an object Mask in parallel with the existing branch for boundary-box recognition [5]. Compared with Faster R-CNN, Mask R-CNN has simple training and lower cost. It is suitable for multitask prediction model, and its integration and comprehensiveness have been enhanced. At present, it has been applied in the field of medical image detection and segmentation to some extent [6]. The architecture of the Mask R-CNN model is shown in Figure 1.

*(1) Backbone*. Backbone is a series of feature maps for extracting images by convolution layer, such as VGG16, VGG19, GooLeNet, ResNet50, and ResNet101. The proposed ResNet (deep residual network) effectively solves the problems of gradient disappearance and gradient explosion caused by the deepening of network layers.

When ResNet is built, the two types of blocks (Identity block and Conv Block) are used interchangeably, as shown in Figures 2(a) and 2(b), respectively.

*(2) Feature Pyramid Network (FPN)*. FPN can distinguish objects of different sizes and different features of objects and use shallow features and depth features to distinguish simple objects from responsible objects. The basic principle is to make use of the characteristics of the convolutional network itself to conduct convolution and pooling operations on images, so as to obtain feature maps of different sizes. Details are emphasized in the shallow network, while semantic information is emphasized in the deep network. The feature extraction process of FPN is shown in Figure 3.

FPN consists of two parts: bottom-up and bottom-up. The bottom-up part realizes the feature extraction function of traditional convolutional network. With the deepening of convolution, the spatial resolution decreases, and the spatial information is gradually lost, but more high-level semantic information can be detected at the same time. In the bottom-up part, the prediction is made according to multiple feature maps [7]. After continuous sampling, the spatial resolution is improved, but the location information of objects is lost at the same time. FPN builds a horizontal link between the reconstructed layer and the feature map so that the detector can better predict the location information of the object, thus replacing the feature extractor in Faster R-CNN and generating a feature pyramid of higher quality.

*(3) Region Proposal Network (RPN)*. RPN outputs various types of rectangular object boxes with scores through images of any scale as input to provide regional proposals. Its architecture is shown in Figure 4.

RPN realizes sliding window processing by using an *N* × *N* window on the feature map output by the shared convolution layer. In each sliding window, multiple region suggestions are realized, that is, *K* anchor boxes, each of which corresponds to an anchor point [8]. For a convolution map of size *W* × *H*, there are a total of *W* × *H* × *K* anchor points.

The loss function of RPN network is defined in

(1) $$\begin{array}{c} L\left(\left\{p_{i}\right\},\left\{t_{i}\right\}\right)=\frac{1}{N_{\text{cls}}}\underset{i}{\sum }L_{\text{cls}}\left(p_{i},p_{i}^{*}\right)+\lambda \frac{1}{N_{\text{reg}}}\underset{i}{\sum }p_{i}^{*}L_{\text{reg}}\left(t_{i},t_{i}^{*}\right), \end{array}$$

where *i* is the index of the anchor points in batch. *p*_*i*_ corresponds to the predicted probability of each anchor point, *p*^∗^ represents the ground truth (GT) tag of training set, *t*_*i*_ represents the vector of parameterized coordinates of anchor boxes, and *t*^∗^ is the vector corresponding to GT bounding boxes.

*(4) Region of Interest (ROI) Align*. ROI Align is based on Faster R-CNN improved by ROI Pooling. After RPN, the model obtains a series of anchor boxes' characteristic values, which are of different sizes and need to be uniformly expressed and input into the full connection layer. In the Faster R-CNN, the ROI Pooling method is used to carry out the Pooling operation in proportion on the original coordinates [9]. Since floating point numbers may appear in the pooling process, it is necessary to carry out the rounding process, so the problem of pixel points not corresponding will be generated. When the feature map is restored to the original image, great errors will be generated, resulting in the loss of feature values. ROI Align uses bilinear interpolation instead of rounding floating-point numbers, which makes the extracted eigenvalues closer to the ROI region of the original image. The accuracy of the mask increases from 10% to 50%, showing a significant effect. The schematic diagram of both is shown in Figure 5.

*(5) Loss Function*. For each ROI, the multitasking loss function is shown in Equation (2) as follows:

(2) $$\begin{array}{c} L=L_{\text{cls}}+L_{\text{box}}+L_{\text{mask}}, \end{array}$$

wherein *L*_cls_ is the classification loss function and *L*_box_ is the regression loss function. The mask branch has *k*∗*m*^2^ dimensions of output for each ROI, that is, binary masks of class *k* resolution *m*^2^. Using a per pixel sigmoid, *L*_mask_ is defined as the average binary cross entropy loss. For ROI belonging to the KTH category, *L*_mask_ only considers the KTH mask, allowing each category to generate masks. Competition between classes is avoided [10].

Through the Faster R-CNN loss function, it can be concluded that the loss function of Mask R-CNN has five parts, including the classification loss function and regression loss function of RPN, and the classification loss function, regression loss function, and mask loss function of ROI. The overall loss function is shown in

(3) $$\begin{array}{c} L_{\text{final}}=L\left(\left\{p_{i}\right\},\left\{t_{i}\right\}\right)+\left(L_{\text{cls}}+L_{\text{box}}+L_{\text{mask}}\right). \end{array}$$

Among them, *L*_mask_ and *L*_box_ only have effects on positive sample ROI.

### 2.2. Mask R-CNN Algorithm for Reusing Underlying Information

The proposed ResNet network effectively solves the problem of gradient disappearance and gradient explosion caused by the deepening of network layers. Its main structure is the stack of multiple residual blocks, namely, identity block and conv block mentioned above. However, despite ResNet's strong learning capability, an excessively deep network still leads to problems with reduced generalization ability, increased number of participants, and longer training time. Therefore, the main architecture of the network is improved by combining two kinds of residual blocks [11]. According to the body of the hip anatomy in X-ray images, the need to identify the main parts including before the iliac spine, pelvis pubic symphysis, big small femur rotor and rotor, such as object is more, so in the backbone network between C1 to C5 layer are stacked to a residual block 4 each residual block includes four convolution layer, eventually making backbone network from top to bottom layer for 42 layer. In order to fit the X-ray image of the training hip joint, the shallower network layer can also prevent the occurrence of overfitting.

This paper implements a multiplexed C1 feature extraction network, as shown in Figure 6. The original image with a size of 640 × 640 × 3 was first input, and the feature image obtained after the first two compressions was defined as C1. Secondly, 256 convolution kernels with step spacing of 1 and size of 3 × 3 were used for convolution operation for C1 to obtain C1C2 with feature graph size of 160 × 160 × 256. Then, P2 was obtained after fusion with C2 unified by channel. For C1, 256 convolution kernels with step spacing of 2 and size of 3 × 3 are used for convolution operation to obtain C1C3 with feature map size of 80 × 80 × 256. After fusion with C3 after channel unification, P3 is obtained. Similarly, 256 convolution kernels with step spacing of 4 and size of 3 × 3 are used for convolution operation for C1 to obtain C1C4, and P4 is obtained after fusion with C4. At this time, the C1 layer has fewer compression times and contains more detailed information, making it easy to detect the lesser trochanter of hip joint. Through this series of steps, the reuse of low-level information is completed, and the detection ability of small objects is improved.

### 2.3. Overall Network Framework

The main architecture of the network is shown in Figure 7.

After the input X-ray image is processed by RPN and local feature layer, the target is identified and segmented. The extracted P2-P6 is used as the input of RPN, in which anchor boxes of different sizes are generated, and the probability of containing specific objects in the area is predicted according to Intersection of Union (IOU), so as to identify bone information of different proportions in the hip joint. The use of RPN is necessary because of the varying size of the hip area to be identified, which makes traditional fixed-length coils difficult to apply.

After obtaining regions of variable size through RPN, ROI Align is utilized to generate output of fixed size. At the same time, the trunk network will input ROI Align to the extracted P2-P6 and determine which layer to map according to the size of the region of interest. The mapping formula [12] is shown in

(4) $$\begin{array}{c} k=\left[k_{0}+lb\left(\frac{\sqrt{xy}}{224}\right)\right]. \end{array}$$

In the formula, *k*_0_ represents the subscripts corresponding to P2-P6 of different scale feature layers, *x* and *y* correspond to the width and height of the region of interest, and *k* is finally obtained by rounded down.

After the ROI Align layer, the network can achieve the feature map of specific dimension size. After that, after a 7 × 7 convolution and a convolution of 1024 × 1 channels used to simulate 1024 full connections, it is connected to the classification and location branches after passing through the full connection layer. At the same time, feature maps of specific dimensions are output through RoI Align layer. Four times of 3 × 3 convolution will be carried out, and then, one deconvolution will be carried out, and then, the number of channels is the number of categories to be identified. Segmentation results will be obtained, and the detection and segmentation function of Mask R-CNN network [13] multiplexed with low-level information is completed.

### 2.4. Experimental Settings

In control group, there were 23 males and 17 females aged from 60 to 80 years. Real-time and routine postoperative rehabilitation nursing guidance for patients, including routine health education, the application of analgesic drugs according to the patient's pain, and as early as possible out of bed activities.

In observation group, there were 20 males and 20 females aged from 60 to 82 years. On the basis of the control group, the algorithm model was used to predict the postoperative recovery of patients. For the possible complications, drugs were used for prevention and control, and surgical treatment was carried out when necessary.

In our paper, we chose four observation indicators. First, the visual analog scale (VAS) represents the pain of the two groups; second, the Harris score represents the recovery of hip joint; third, the Barthel index represents patients' self-care ability; last, the incidence of complications, including anemia, infection, and stress injury. We will compare the above indicators between control group and observation group to evaluate the recovery condition of these patients.

Finally, SPSS 22.0 statistical software was used to process the data. Measurement data were expressed as *X* ± *S*, *t* test was used, count data were expressed as percentage, *χ*^2^ test was performed, *P* < 0.05 meant that the difference was statistically significant.

### 2.5. Classification and Screening of Hip Joint Image Data

According to the FAI concept proposed by Ganz et al. [14], complications after hip replacement can be roughly divided into four types, namely, no disease, Cam collision type, Pincer collision type, and mixed type. The medical characteristics and comparison with normal hip joint X-ray images are shown in Figure 8.

Cam-type: the direct manifestations were bony protuberance of the anterior upper margin of the femoral head and neck junction, insufficient intercervical depression of the femoral head, accompanied by local hyperosteogeny, that is, “left hand handle” deformity; nonspherical changes of femoral head; femoral head and neck eccentricity decreased; the femoral neck angle (A angle) increased. These lesions are likely to lead to degenerative changes in the hip, resulting in the formation of acetabular margin osteophytes or free calcification. For this lesion type, the key of classification lies in identifying the size of angle A, and angle A > 50° is the critical value for judging this type of FAI lesion, as shown in Figure 9(a).

Pincer-type: direct manifestations of acetabular dysplasia, including acetabular depth, acetabular tilt forward, acetabular tilt back, acetabular posterior wall overcoverage; secondary degenerative changes of the hip, including acetabular margin ossification or calcification; joint space narrowed and joint surface capsule changed. Cystic changes in the anterior upper margin of femoral neck and thickening of adjacent bone cortex. Such lesions can easily lead to deformation or displacement of the acetabulum and then acetabular labial ossification. For this type of lesion, the key to classification is to identify the LCE angle at the central margin (the center of the femoral head is defined as point C, and the sclerotic band below the acetabular margin is defined as point E for external aid). The LCE angle < 20° can be diagnosed as hip dysplasia, and >39° can be diagnosed as acetabular overcoverage, as shown in Figure 9(b).

Mixed-type: Cam-type and Pincer-type rarely occur independently, and mixed-type is the case when the two types occur simultaneously. Mixed-type has two types of hip joint morphological characteristics at the same time. Therefore, if the target has both Cam-type characteristics and Pincer-type characteristics, it can be diagnosed as mixed-type.

According to FAI classification, hip joint images of patients were divided into four categories in this paper, namely, normal, CAM-type, Pincer-type, and mixed-type. In order to effectively judge the type and degree of disease in patients, a large number of comparative experiments were conducted in this paper. 7132 hip joint images were used, and the data of poor quality were excluded by preprocessing. Exclusion criteria: ① patients with other fractures; ② patients with coagulation dysfunction; ③ patients with dysfunction of important organs; ④ before the onset of motor dysfunction [15]. A total of 3500 pieces of experimental data were obtained, as shown in Table 1 and Figure 10.

## 3. Results

### 3.1. Hip Imaging Data Preprocessing

By observing the number of samples, we found that nearly half of the patients in all samples belonged to the type without disease. Among the samples with disease, the mixed type was the main type, and the proportion of Cam type and Pincer type was very small. There was a large difference in the number among all samples. We believe that, in the prediction results of the model, more attention should be paid to correctly predicting the types of latent complications, rather than to learning the medical image features of unaffected patients. Therefore, we should undersample the medical samples of normal patients with edit nearest neighbor (ENN) [16] and through traversing most types of samples. If most of its *K*-nearest neighbor samples are different from their own categories, we delete them to reduce the impact of data imbalance on the predicted results. At the same time, according to the clinical needs, a binary model was set up to detect whether patients have disease.

In order to avoid the problem of overfitting the training samples and improve the generalization ability of the model, according to the characteristics of the training samples, this paper divides the training set and the test set by the method of cross validation of tenfold. First of all, the original data set is divided into equal tenfold. In each compromise, the proportion of different types of data is the same as that of the original data, so as to avoid the loss of certain types of data. In each iteration, one fold was successively selected as the test set and the remaining data as the training set to ensure that the training set and test set were independent of each other. This was repeated for ten times, and the average accuracy rate was taken as the final accuracy rate of the model.

### 3.2. Clinical Verifications

VAS scores of the two groups were compared in Table 2.

Harris hip scores before and after intervention were shown in Table 3.

Barthel scores of the two groups before and after intervention were compared in Table 4.

The complications of the two groups were compared in Table 5.

The results show that deep learning-based nursing model of hip surgery can accurately evaluate the postoperative situation of patients and timely predict and treat potential complications. By comparison, patients in the control group had more mild postoperative pain, higher Harris score and Barthel score, and lower incidence of postoperative complications. The difference was statistically significant through the test of statistical principle.

## 4. Discussion

At present, postoperative rehabilitation of patients after THA in China is still carried out in the traditional way of nursing. When designing the nursing plan, experienced physicians are required to observe the patients, and the process is complicated and susceptible to subjective factors [17]. The quality of life of patients after hip replacement is seriously affected by different surgical results, physiological conditions, and living habits of patients, resulting in a high incidence of complications.

In clinical applications, X-ray films have been shown to be useful in predicting potential complications in patients. However, due to lack of experience, and evaluation results are prone to observation error of attending physicians, the effect is not very ideal.

Besides, deep learning has been applied in various medical fields, but in postoperative care, there are few related applications, which are still in the exploratory stage.

In this paper, deep learning is applied in the field of postoperative nursing of hip joint. Mask R-CNN model is used to provide postoperative nursing advice and guidance for doctors by using patients' hip X-ray images. After clinical trial comparison, the effect is significant.

## 5. Conclusion

This paper summarizes the hip replacement cases in recent years, and designs the Mask R-CNN deep learning model based on X-ray images. In this paper, the prosthetic matching accuracy of patients was analyzed by segmentation and identification of hip X-ray images. At the same time, FAI classification was used to classify the patient's recovery, predict the possible types of complications, and provide nursing advice. The model achieved good performance through the training of a large number of medical case images. In clinical trials, the observation group and the control group were evaluated by VAS score, Harris and Barthel index, and complication rate. The experimental results showed that patients in the observation group were better than those in the control group in terms of pain, hip joint ability score, self-care ability, and complication rate, and the difference was statistically significant through the calculation of statistical principles. Therefore, it is a feasible attempt to apply deep learning method to postoperative nursing of patients undergoing hip replacement surgery, with high clinical application potential.

## Figures and Tables

**Figure 1:** Mask R-CNN network architecture.

**Figure 2:** ResNet framework based on (a) identity block and (b) conv block.

**Figure 3:** FPN feature extraction process.

**Figure 4:** RPN architecture.

**Figure 5:** ROI pooling compared to ROI Align.

**Figure 6:** Reuse C1 layer feature extraction network.

**Figure 7:** Improved Mask R-CNN process.

**Figure 8:** Image comparison of different types of hip joint.

**Figure 9:** Classification and screening of hip joint based on (a) femoral neck angle and (b) LCE angle.

**Figure 10:** X-ray film samples.

**Table 1:** Statistical table of hip joint image samples.

Type	Sample size	Proportion	Label 1
Nondisease	1789	51%	1
Cam-type	209	6%	2
Pincer-type	203	6%	3
Mixed type	1299	37%	4

**Table 2:** VAS scores comparison.

Items	Observation group	Control group
Admission date	4.01 ± 2.10	4.29 ± 2.77
Postoperation day	2.29 ± 0.92	4.12 ± 1.10
7 days after operation	1.17 ± 0.28	3.05 ± 0.33

**Table 3:** Harris scores comparison.

Group	Before intervention	After intervention
Observation group	46.75 ± 5.41	79.47 ± 4.20
Control group	46.87 ± 5.37	67.26 ± 4.16
*t* value	0.067	13.017
*P* value	0.948	0.001

**Table 4:** Barthel scores comparison.

Group	Before intervention	After intervention
Observation group	44.62 ± 4.40	76.34 ± 3.15
Control group	44.70 ± 4.88	62.65 ± 3.98
*t* value	0.105	17.092
*P* value	0.916	0.001

**Table 5:** Complication comparison.

Group	Anemia	Infection	Pressure injury	Overall rate
Observation group	1	0	0	2.5%
Control group	1	2	1	10.0%
*χ* ^2^ value				5.17
*P* value				0.023

## Data Availability

Data are available on request from the authors due to privacy/ethical restrictions.
